# The Construction and Effect Analysis of Nursing Safety Quality Management Based on Data Mining

**DOI:** 10.1155/2022/6560452

**Published:** 2022-06-02

**Authors:** Yimei Yang, YanHong Deng, Haimei Zhang

**Affiliations:** ^1^Central Sterile Supply Department, Chongqing University Cancer Hospital, Chongqing 400030, China; ^2^Department of Neuro-Oncology, Chongqing University Cancer Hospital, Chongqing 400030, China; ^3^Department of Urologic Oncology, Chongqing University Cancer Hospital, Chongqing 400030, China

## Abstract

Data mining belongs to knowledge discovery, which is the process of revealing hidden, unknown, and valuable information from a large amount of fuzzy application data. The potential information revealed by data mining can help decision-makers adjust market strategies and reduce market risks. The information mined can be the discovery of a particular study and little known, which must be based on the principle of truth. Nursing safety means that during nursing work, the nursing staff must strictly follow the nursing system and operating procedures, accurately execute doctor's orders, implement nursing plans, and ensure that patients get physical and mental safety during treatment and recovery. This paper aims to explore the construction of nursing safety quality management system and its effect analysis based on data mining. It is hoped that improvements in hospital nursing processes will provide better nursing services for patients using data mining techniques. This paper uses the FP algorithm to mine the data set and generates frequent itemsets, proposes and implements the association rule mining algorithm, and obtains the association rules with practical reference value. This article analyzes the current status and existing problems of nursing management, and puts forward some problems existing in the current nursing management staff's own quality, nursing quality system standards, and nursing management system. The experimental results in this article show that there are 42 cases of poor nursing due to lack of basic medical knowledge, accounting for 52%; there are 12 cases of poor nursing due to their own diseases, accounting for 15%; there were 7 cases of poor nursing due to lack of communication, accounting for 9%; there were 15 cases of poor nursing caused by unreasonable use of restraint devices, accounting for 19%. From these data, it can be seen that patients need to have basic medical knowledge and act in strict accordance with doctors' orders. Family members also need to accompany the patients more and cooperate with all parties in order to maximize the effectiveness of care.

## 1. Introduction

With the development and popularization of modern information technology, the amount of data in society is increasing exponentially. In the early stages of development, it can indeed help us obtain massive amounts of information and keep abreast of the situation. However, IoT technology has triggered a flood of information in the 21st century due to its successful application in the field of production. How to find the required information within the scope of the massive information has become an urgent problem to be solved. How to mine the valuable information hidden behind the massive information has also become a current research hotspot. Although traditional databases can collect and query information, they cannot analyze the underlying rules behind the information and cannot make predictions for future development. In order to solve this problem in the future, data mining came into being. The deepening reform of economic policies has also led to the development of the medical industry. However, in recent years, the doctor-patient relationship has gradually deteriorated and disputes have continued. The patient's demand for nursing services is increasing, and the workload of the nursing staff is also increasing, resulting in the failure of real and effective improvement in nursing work. To this end, we combine data mining technology with nursing work, apply modern science and technology to various fields of the nursing industry, further explore new nursing methods, improve the quality of nursing, ease the relationship between doctors and patients, and promote the progress of medical care.

Nursing work is an important part of medical and health work. Improving the level of care can effectively alleviate the relationship between doctors and patients and improve the quality of medical care. The quality of nursing work is one of the important indicators of the quality of hospital medical services, which is directly related to the medical safety, treatment effect, and physical recovery of patients. This is an effective measure to improve the level of nursing, which can not only improve the treatment effect but also promote the development of the nursing industry.

Data mining technology can analyze the information hidden in the data, provide a theoretical basis for business decisions, improve the governance capabilities of government departments, and reduce unnecessary losses. Combining data mining technology with nursing care can provide patient information in time, reduce unnecessary friction, and build a good doctor-patient relationship. Yan and Zheng constructed a “universe” containing more than 18,000 fundamental signals from financial statements, and used guided methods to evaluate the impact of data mining on fundamental anomalies. He found that even after considering data mining, many fundamental signals are important predictors of cross-sectional stock returns. This predictive ability is more pronounced after periods of high sentiment and in stocks with greater arbitrage restrictions. Experimental evidence shows that fundamental anomalies, including those newly discovered in research, cannot be attributed to random chance, and mispricing can better explain them [1]. In order to deal with the dynamics of training samples and improve the prediction accuracy, Wu and Peng proposed a short-term WPF data mining method consisting of K-means clustering and bagging neural network (NN). Based on the similarity between historical days, K-means clustering is used to divide the samples into several categories, which contain weather condition information and historical power data. In order to overcome the over-fitting and instability problems of traditional networks, he integrated the integration method into the back-propagation neural network. In order to confirm the validity, the proposed data mining method was checked on the real wind power data trajectory. The simulation results show that compared with other baselines and existing short-term WPF methods, it can obtain better prediction accuracy [2]. Some Scholars focus on the methods of quality management in the nursing department by implementing continuous improvement cycles, improving team participation, monitoring systems, and external evaluation quality models (EFQM, ISO). The key to the correct implementation of the quality management system is to obtain the support of the health facility manager, because the manager is responsible for designing the action strategies involved in the quality management system and communicating it to the health professionals. The implementation of the quality management system will minimize or eliminate preventable adverse effects and promote patient safety and safety practices for health professionals [3]. In order to conduct research on health care reporting, Blenkinsopp et al. not only provided valuable insights on the factors affecting health care reporting and how organizations responded but also found a huge gap in the coverage of the literature on over-focusing on care, and focused on the early stages of the reporting process. This review identified gaps in the reported literature in health care. Although there are limitations, it can determine the importance of practice, including enhancing employees' sense of security and providing ethical training [4]. Ramos et al. proposed a framework based on data mining technology and adjusted for selection, which is a new hybrid framework with gene subsets of target diseases performed in DNA microarray experiments. The framework involves methods such as statistical significance testing, cluster analysis, evolutionary computation, visual analysis, and boundary points. Another novelty of this work is that the patient's age is used as an additional factor in the analysis, which can give us a deeper understanding of the disease [5]. Lin et al. proposed the use of human behavior modeling and data mining to predict human error, because it also uses top-down reasoning to transform the interaction between task features and conditions into a general tendency for operators to make mistakes. And bottom-up analysis interprets the psychophysiological measurement results as the possibility of individuals making mistakes on a trial-by-trial basis. This linear discriminant analysis can improve classification performance by combining real-time electroencephalographic (EEG) features acquired in digital typing experiments with modeled features generated by an enhanced human behavior model (a queuing network model human processor) [6]. Yang et al. proposes a faster way to detect potential failures by identifying possible variables that lead to failures at specific times. The method he proposed uses data mining technology to select more important variables from the turbine monitoring and data acquisition (SCADA) system to improve prediction accuracy, and use the control chart based on the exponentially weighted moving average (EWMA) model to implement the residual method to eliminate the autocorrelation in the data. Both EWMA and multivariate EWMA (MEWMA) control charts are constructed to compare their detection capabilities and the types of errors generated. Experiments prove that the method is effective [7]. Although these theories have explored data mining technology and nursing safety management to a certain extent, the correlation between the two is not enough to produce results in application.

In the process of exploration, this article uses the existing industry rules as the theoretical basis, and the quality and safety evaluation indicators are well-founded, avoiding the inconsistency of the exploration indicators with reality. This article introduces the amount of nursing care into the management of nursing safety and quality for the first time, analyzes the quality and quantity of nursing work, and improves the enthusiasm of nursing work. This article explores family nursing and provides a basis for constructing a comprehensive nursing safety and quality management system.

## 2. The Construction and Effect Analysis Method of Nursing Safety Quality Management Based on Data Mining

### 2.1. Overview of Data Mining

Data mining refers to the application of data mining technology to a very large amount of irregular data, so as to obtain hidden information that is beneficial to value [8]. In fact, data mining is the result of the gradual evolution of information technology. In recent years, the rapid development of the Internet of Things technology has made it widely used in the field of social production. In particular, the advancement of Internet technology has become a necessary means for enterprises to construct information systems [9]. The analysis of Internet engines in the era of big data is shown in Figure 1:

It is a research hotspot to obtain the most effective information based on the massive database in the shortest time during this era of knowledge economy. Data mining technology can find the key information from the massive information and obtain the potential value of the information [10, 11].  Figure 2 is a specific data mining flowchart:

From the perspective of the work source of data mining technology, data mining is mainly a process of extracting and utilizing potentially valuable information in massive amounts of information [12]. Data mining technology has gone through four steps: data collection, data access, data warehouse, and data mining. The mining process of data mining is shown in Figure 3:

In the contemporary era of highly developed information technology, data mining is not only satisfied with query and storage, but it is more important to use information to assist decision-making, and the data warehouse mentioned above can well complete the auxiliary decision-making work. As a data collection place, the data warehouse can make reasonable use of data analysis technology to obtain the required information from the massive amount of information. The data warehouse includes three structures: data collection, data storage, and data access. These three structures cooperate with each other to analyze and process data to meet the decision-making needs in enterprise management [13, 14]. The system structure of the data warehouse is shown in Figure 4:

The most important thing in the entire data mining process is to establish a data warehouse. After determining the scope of the information, it needs to choose a suitable data analysis tool [15]. How to choose data mining technology needs to consider the difference of the data and combine the characteristics of the data. In fact, when the data mining results are presented, they may not meet the actual needs, which require the results to be analyzed again. If it is found that the structure is indeed contradictory after analysis, then it is necessary to re-select the information range and re-analyze with new mining techniques until the result meets expectations [16, 17]. The calculation process is shown in Figure 5:

### 2.2. Data Mining Algorithm

The decision tree is essentially the process of classifying and analyzing data. Its analysis process appears in a tree-like form, and each node represents a different type of data [18]. The specific structure is shown in Figure 6:

Traditional information expression has uncertainty. We express this uncertainty as:

(1) $$\begin{array}{c} W\left(A\right)=f\left(a_{1}\right)j\left(a_{1}\right)+f\left(a_{2}\right)j\left(a_{2}\right)+\cdots +f\left(a_{l}\right)j\left(a_{l}\right)=-\sum_{k}^{l}f\left(a_{k}\right)\log_{2}\;F\left(a_{k}\right). \end{array}$$

When *f*(*a*_1_)=*f*(*a*_2_), *W*(*A*)=1.

(2) $$\begin{array}{c} j\left(f,k\right)=-\frac{f}{f+k}\log_{2}\frac{f}{f+k}-\frac{k}{f+k}\log_{2}\frac{k}{f+k}. \end{array}$$

Formula (2) represents the amount of information required for the correct classification of the decision tree.

(3) $$\begin{array}{c} Y\left(B\right)=\sum_{K}^{s}\frac{f_{k}+l_{k}}{f+l}j\left(f_{k},l_{k}\right). \end{array}$$

Among them, *B* represents a subset of the function decision tree, *j* represents the information expectation, and *Y*(*B*) represents the average value of the information expectation.

(4) $$\begin{array}{c} \text{gain}\left(B\right)=J\left(f,l\right)-Y\left(B\right), \end{array}$$

gain(*B*) represents the information gain with attribute *B*.

(5) $$\begin{array}{c} J\left(c_{s}\right)=-\sum_{k}^{x}f_{k}\log_{2}\left(f_{k}\right). \end{array}$$

Among them, *c*_*s*_ represents the subset, and *J* represents the amount of information in the subset.

(6) $$\begin{array}{c} Y\left(B\right)=\sum_{h}^{s}\frac{\left|c_{s}\right|}{\left|g\right|}*J\left(c_{s}\right). \end{array}$$

*Y*(*B*) represents the information expectation required when *B* is the attribute.

(7) $$\begin{array}{c} \text{Gain Ratio}\left(D\right)=\frac{\text{Gain}\left(B\right)}{\text{Split }I\left(B\right)}. \end{array}$$

Formula (7) is a functional expression of gain ratio, which can eliminate the drawbacks caused by information gain.

(8) $$\begin{array}{c} \text{Split }I\left(Q\right)=-\sum_{f}^{s}\frac{\left|c_{s}\right|}{G}*\log_{2}\left(\frac{\left|c_{s}\right|}{G}\right), \end{array}$$

where Split *I*(*Q*) represents split information.

(9) $$\begin{array}{c} W=\sum_{k}^{n}\frac{g_{k}}{G}\log_{2}\frac{g_{k}}{G}, \end{array}$$

where *G* stands for sample data, and *g* stands for quantity.

(10) $$\begin{array}{c} W_{1}=\frac{G_{1}}{G}\left(-\frac{G_{2}}{G_{1}}\log_{2}\frac{G_{2}}{G_{1}}\right). \end{array}$$

Formula (10) represents the information entropy when the sample data is 1.

(11) $$\begin{array}{c} W_{2}=\frac{G_{3}}{G}\left(-\sum_{k}^{n}\frac{G_{3i}}{G_{3}}\log_{2}\frac{G_{3i}}{G_{3}}\right). \end{array}$$

Among them, 3*i* represents the number of classifications. The approximate information gain value at this time is:

(12) $$\begin{array}{c} \text{Gain}\left(p\right)=W-W_{1}-W_{3}=-\sum_{K}^{m}\frac{g_{k}}{G}\log_{2}\left(\frac{g_{k}}{G}\right)\left(\frac{g_{1}}{G}\right)\left(-\frac{G_{2}}{G_{1}}\log_{2}\frac{G_{2}}{G_{1}}\right). \end{array}$$

When the obtained value is greater than zero, it is retained, if it is less than zero, it is not retained.

(13) $$\begin{array}{c} W\left(Q\right)=-\frac{c}{c+v}\log_{2}\frac{c}{c+v}-\frac{v}{c+v}\log_{2}\frac{v}{c+v}, \end{array}$$

*c*, *v* represent the two attributes of the data set.

(14) $$\begin{array}{c} T\left(Q_{j}\right)=-\frac{c_{j}}{c_{j}+v_{j}}\log_{2}\frac{c_{j}}{c_{j}+v_{j}}-\frac{v_{j}}{c_{j}+v_{j}}\log_{2}\frac{v_{j}}{c_{j}+v_{j}}. \end{array}$$

*T*(*Q*_*j*_) represents the expected information of the data subset.

(15) $$\begin{array}{c} W\left(Q_{j}\right)=\sum_{j}^{s}\frac{c_{j}+v_{j}}{c+m}T\left(Q_{j}\right)=\frac{1}{\left(c+v\right)}\sum_{j}^{s}\left(-c_{j}\ln\frac{c_{j}}{c_{j}+v_{j}}-v_{j}\ln\frac{v_{j}}{c_{j}+v_{j}}\right). \end{array}$$

Formula (15) represents the calculation formula of information entropy.

(16) $$\begin{array}{c} \ln\left(1+m\right)=\sum_{l}^{\infty }\frac{{\left(-1\right)}^{l+1}}{l!}m^{l}. \end{array}$$

Formula (16) represents the expression of McLaren series function.

(17) $$\begin{array}{c} \ln\left(1+m\right)=\sum_{l}^{\infty }\frac{{\left(-1\right)}^{l+1}}{l!}m^{l}=m. \end{array}$$

When *m*⟶−*∞*, it can simplify formula (16) to formula (17).

(18) $$\begin{array}{c} W\left(Q\right)=-\frac{c}{c+v}\log_{2}\frac{c}{c+v}-\frac{v}{c+v}\log_{2}\frac{v}{c+v}=\frac{2}{\ln\;2}\frac{cv}{{\left(c+v\right)}^{2}}. \end{array}$$

Substituting formula (17) into formula (13) can obtain simplified function expression (18).

(19) $$\begin{array}{c} T\left(Q_{j}\right)=\frac{1}{\left(c+v\right)}\sum_{j}^{s}\left(-c_{j}\ln\frac{c_{j}}{c_{j}+v_{j}}-v_{j}\ln\frac{v_{j}}{c_{j}+v_{j}}\right)=\sum_{j}^{s}\frac{2c_{j}v_{j}}{v_{j}+c_{j}}. \end{array}$$

Substituting formula (17) into formula (15) can obtain simplified function expression (19).

(20) $$\begin{array}{c} L\left(Q_{j}\right)=-c_{j}\log_{2}\frac{c_{j}}{c_{j}+v_{j}}+v_{j}\log_{2}\frac{v_{j}}{c_{j}+v_{j}}=\frac{2}{\ln\;2}\frac{c_{j}v_{j}}{{\left(c_{j}+v_{j}\right)}^{2}}. \end{array}$$

*L*(*Q*_*j*_) represents information measurement.

### 2.3. Nursing Safety and Quality Management

With the improvement of living standards, the reform of the medical system is inevitable [19]. As the society pays more attention to “people,” people's requirements for nursing services are getting higher and higher. The development of modern science and technology has made the medical field more advanced, and the combination of modern technology and the medical industry has provided nursing work more room for improvement [20, 21]. The nursing department is a special department in the medical field. Although it serves various departments, it is not affiliated with any department. Nursing work occupies a very important position in the whole medical process, which not only affects the medical effect but also affects the overall image of the hospital. Although the current level of nursing care is relatively high, there are still many shortcomings in nursing management, such as the current sensitive doctor-patient relationship and medical disputes [22, 23].

The definition of nursing was first proposed by the American Nursing Association, which believes that nursing is a response to existing health problems. Nursing is a comprehensive subject, based on natural subjects and social subjects. Some scholars attempt to improve nursing management by exploring the theoretical knowledge of maintaining and restoring human health [24, 25].

Nursing management is subordinate to management and aims to improve management level and management efficiency [26]. Nursing management plays an important role in the whole benefit arrangement and diagnosis process. The proportion of the nursing staff in hospitals has exceeded 30%, and it has been increasing, while the nursing staff can directly participate in and manage more than 70%. From this data point of view, the work quality of the nursing staff directly affects the work quality of the entire medical care [27, 28].

## 3. The Construction and Effect Analysis Experiment Based on Data Mining in Nursing Safety Quality Management

### 3.1. Object

In this experiment, a sampling survey method was adopted to investigate the nursing staff in a tertiary hospital in Chongqing, and the nursing quality was discussed according to the nursing time and education of the nursing staff.

According to the data in Table 1, this experiment investigated the basic conditions of 20 nursing workers, who were widely distributed, roughly between 28 and 44 years old. According to the nursing age and job title, the longer the nursing job and the richer the work experience, the higher the job title. The head nurses of this hospital generally take longer to care for. In terms of academic qualifications, the nursing staff mainly have a bachelor's degree, and a graduate degree is less. According to the job distribution of nursing staff, the workers with longer nursing time are concentrated in the emergency department and operating room, and the nursing workers with less experience are concentrated in the conventional ward.

According to the data in Table 2, in addition to investigating the primary care situation of a tertiary hospital in Chongqing, we also have a brief understanding of the composition of the hospital's experts. According to the survey, the experts have worked for more than 10 years, and they are mainly doctors, which prevents the shortcomings of insufficient experience and insufficient level. Moreover, the professional fields of these experts are mainly medical management and nursing management, and they are related to the subject of this investigation, which ensures the validity of the data.

### 3.2. Experimental Method

In this experiment, a questionnaire survey was used to investigate the overall quality of care in a tertiary hospital in Chongqing. Before issuing the questionnaire, we explained to the hospital staff and explained the purpose and requirements of investigation to make the results as scientific and true as possible. In this experiment, 200 questionnaires were distributed, and 145 questionnaires were returned, with an effective rate of 72.5%.

According to the data in Table 3, there are many reasons for the low quality of care. We have cited several types of common adverse nursing events. Among them, there were 16 cases of poor nursing caused by errors in nursing text records, accounting for 11%. There were 10 cases of poor nursing caused by drug sensitivity errors, accounting for 7%; there were 7 cases of poor nursing caused by interns alone, accounting for 5%. There were 40 cases of poor nursing caused by slippage of the pipeline, accounting for 27%; there were 37 cases of poor nursing caused by other events, accounting for 26%. Slippage of the pipeline is most likely to cause nursing errors. Therefore, this type of operation training should be strengthened in the usual training process to reduce errors and improve the quality of care.

### 3.3. Factors Related to the Quality of Nursing Safety Management

According to the nursing adverse events outlined above, it is found that there are many reasons for the low quality of care, which may be caused by the mistakes of the nursing staff, or it may be due to the patient's own reasons.

According to the data in Table 4, it was found in the process of nursing safety and quality management survey that there were 86 cases of poor nursing due to nursing operation errors, accounting for 59%. There were 39 cases of poor nursing conditions caused by patients' own factors, accounting for 27%; there were 10 cases of poor nursing cases caused by environmental factors, accounting for 7%. There were 3 cases of poor nursing caused by equipment, accounting for 2%; there were 3 cases of poor nursing caused by medical equipment, accounting for 2%. There were 4 cases of poor nursing care caused by other reasons, accounting for 3%. Among the overall related factors, nursing operation errors accounted for the highest proportion of poor nursing care, indicating that the nursing staff should strengthen training, improve practical skills, and reduce errors.

In order to investigate the satisfaction level of nursing care in hospitals, a questionnaire survey was conducted on the basis of data mining techniques, as shown below.

Based on the data in Table 5, it is clear that care in this hospital is relatively good overall, but there is room for strengthening in terms of explaining precautions, medication, and diet for patients with high fever.

## 4. The Construction and Effect Analysis of Nursing Safety Quality Management Based on Data Mining

### 4.1. Causes of Poor Care

In the experimental part, the reasons for the poor nursing situation are discussed. Generally speaking, the most important ones are the nursing staff and the patients themselves. In order to improve the quality of care, we conducted a detailed analysis of the causes of the nursing staff's errors and the causes of patients, and looked for solutions for different causes.

The results in Figure 7 show that patients and caregivers were discussed separately when discussing the causes of poor nursing care. The picture on the left shows the operation status of the nursing staff. According to the survey data, there are 65 cases of poor nursing caused by insufficient assessment by the nursing staff, accounting for 45%; 33 cases of poor nursing caused by lack of strict inspection by the nursing staff, accounting for 23%. There were 18 cases of poor nursing caused by lack of basic nursing knowledge of the nursing staff, accounting for 12%; and 25 cases of poor nursing caused by lack of service awareness of the nursing staff, accounting for 17%. There were 4 cases of bad nursing caused by the nursing staff's illegal operation, accounting for 3%. It can be seen that the nursing staff accounted for the highest proportion of cases due to insufficient assessment based on this analysis. This requires the nursing staff to take scientific and effective measures in a timely manner by improving their ability to judge in the face of complex nursing situations. The lack of strict inspection by the nursing staff is also an important reason for poor nursing. This requires the relevant departments of the hospital to formulate corresponding systems to punish the lack of strict inspection and curb the occurrence of such unfavorable situations. As a special service industry in the nursing industry, it is a positive and effective measure to strengthen the training of the nursing staff to avoid mistakes due to lack of nursing knowledge. Treating patients requires the necessary service spirit, provide corresponding services in strict accordance with industry specifications, and strictly prohibit illegal operations [29, 30].

The picture on the right shows poor nursing care caused by patients themselves. According to survey data, there are 42 cases of poor nursing care caused by patients' lack of basic medical knowledge, accounting for 52%. There were 12 cases of poor nursing due to their own diseases, accounting for 15%; there were 7 cases of poor nursing due to lack of communication, accounting for 9%. There were 15 cases of poor nursing caused by improper use of restraint devices, accounting for 19%. There were 4 cases of poor nursing due to lack of companionship, accounting for 5%. From this data, it can be seen that patients need basic medical knowledge, act in strict accordance with medical advice, and actively communicate with medical staff for situations that they do not understand. Family members also need to accompany patients more and cooperate with multiple parties to maximize care.

According to the data in Figure 8, there are many factors that affect the society's management of nursing safety and quality, but they mainly include practical experience, theoretical analysis, reference literature, and intuitive perception. A survey conducted with authoritative experts from a tertiary hospital in Chongqing found that 15 people think that practical experience is very important, 8 people think that practical experience is not very important, and 5 people think that practical experience is not important. There are 7 people who think that theoretical analysis is very important, 5 people think that theoretical analysis is not very important, and 12 people think that theoretical analysis is not important. There are 3 people who think that the amount of literature storage is very important, 5 people who think that the amount of literature storage is not very important, and 7 people who think that the amount of literature storage is not important. There are 8 people who think that intuitive feeling is very important, 7 people who think that intuitive feeling is not very important, and 9 people who think that intuitive feeling is not important. From these data, it can be seen that different medical departments have different degrees of recognition of the four elements, but it is a consensus that practice is very important. Therefore, medical staff should improve their practical ability.

### 4.2. Knowledge of Safety Management of the Nursing Staff

The construction of nursing safety management quality requires a certain degree of nursing safety management knowledge. In this experiment, a survey was conducted based on the current safety management knowledge of medical staff in a tertiary hospital in Chongqing, and a brief analysis of the management of a tertiary hospital in Chongqing was conducted.

According to the data in Figure 9, it is found that the overall level of a tertiary hospital in Chongqing is very average through a survey of nursing safety management knowledge. According to the survey data, the frequency of meetings held within the hospital is 4 points, with a full score of 10 points, accounting for 40%. Generally speaking, the frequency of meetings is not much, and the overall effect is poor. The total number of bad nursing in the hospital was 3.7 points, with a perfect score of 10, accounting for 37%. The overall satisfaction of the nursing effect is low, and the hospital needs to strengthen the training of the nursing staff. The hospital's internal quality scored 4.6 points, accounting for 46%. These data show that the effectiveness of nursing management is insufficient and there is still a lot of room for improvement. The hospital's nursing safety management score is 5.6, accounting for 56% of the total score. These data show that the nursing staff have a general grasp of nursing knowledge and lack of attention to nursing knowledge. The hospital's medical record document writing scored 6 points, accounting for 60% of the total score. These data show that the medical record writing is relatively standardized, but the details are still insufficient. The hospital quality inspection frequency is 7.1 points, accounting for 71% of the total score. These data show that the hospital has a large number of inspections, which is helpful to improve the overall quality of the hospital. The nursing staff scored 6.9 points for their knowledge of medicines; these data show that the nursing staff are not familiar with medicines and are likely to cause work errors.

### 4.3. Nursing Safety Management Knowledge Training

The knowledge of nursing safety management is of great significance to improve the quality of hospital care. This time, a brief analysis is carried out on the nursing safety management knowledge training of a tertiary hospital in Chongqing.

According to the data in Figure 10, there are 40 nursing staff who do not know the difference between nursing disputes, nursing shortcomings, and nursing accidents. There are 72 nursing staff who have not been trained on nursing disputes, nursing shortcomings, and nursing accidents, and 9 who have started training but have forgotten. These data shows that hospitals pay less attention to nursing accidents, which leads to some nursing staff taking up their posts without professional training. This requires the hospital to carry out relevant training regularly to solve the knowledge blind spots and improve the quality of care. The results showed that 27 nurses did not know how to regulate patient medication, 77 nurses did not receive training on regulating patient medication, and 5 forgot the training content. These data show that the hospital's medication is not standardized and the relevant training is insufficient. There are 19 people who do not know how to keep and use medicines, 65 people who have not been trained to keep and use medicines, and 16 people who have forgotten after training. These data show that the hospital did not meet the training requirements. Judging from the critical situation report process, 13 people did not understand the situation, 39 people did not undergo the critical situation report process training, and 25 people forgot after the training. These data show that the emergency response capability of the hospital needs to be improved, and the emergency response process training needs to be strengthened. According to the investigation of patients' suicide or wounding, there are only 13 people who have not received special training, indicating that the hospital is well trained in emergency rescue. From the point of view of the emergency response party for drug loss, only 11 people did not know the treatment process, and 23 people did not participate in the training. These data show that the drug treatment situation is not comprehensive enough. From the overall results of the survey, hospitals need to strengthen relevant training on nursing safety management knowledge.

## 5. Conclusions

The progress of science and technology has accelerated the process of social development. In order to adapt to the development of society, the industry must undergo changes. As the public pays more attention to health, how to improve the quality of care has become the focus of current research. This article aims to study the construction and effect analysis of nursing safety quality management based on data mining, and hopes to use data mining technology to explore the improvement of hospital nursing process and provide patients with better nursing services. Although the article analyzes nursing quality management, there are still shortcomings: (1) There are many types of patients, and how to formulate different care models according to different patients has not been considered. (2) The data source is single, the information is not comprehensive, and the results of the analysis have limitations.

## Figures and Tables

**Figure 1:** Analysis graph of Internet engine results.

**Figure 2:** Data mining flowchart.

**Figure 3:** Data mining process.

**Figure 4:** The system structure of the data warehouse.

**Figure 5:** Data mining process.

**Figure 6:** Decision tree structure.

**Figure 7:** Analysis of the main reasons for poor nursing.

**Figure 8:** Factors affecting nursing quality and safety management.

**Figure 9:** Knowledge of nursing safety management.

**Figure 10:** Nursing safety management knowledge training.

**Table 1:** Subject's information.

Object	Age protection	Age	Position	Academic qualifications	Positions

1	15	40	Head nurse	Undergraduate	Emergency nurse
2	20	43	Head nurse	Undergraduate	Surgical nurse
3	17	37	Head nurse	Postgraduate	Ward nurse
4	19	39	Head nurse	Postgraduate	Surgical nurse
5	5	30	Nurse	Undergraduate	Ward nurse
6	3	28	Nurse	Undergraduate	Ward nurse
7	13	29	Nurse	Postgraduate	Ward nurse
8	7	28	Nurse	Postgraduate	Emergency nurse
9	9	41	Nurse	Undergraduate	Surgical nurse
10	15	44	Head nurse	Undergraduate	Ward nurse
11	7	39	Head nurse	Undergraduate	Surgical nurse
12	5	31	Nurse	Undergraduate	Emergency nurse
13	9	29	Nurse	Postgraduate	Surgical nurse
14	17	33	Nurse	Undergraduate	Ward nurse
15	6	37	Head nurse	Undergraduate	Emergency nurse
16	10	32	Nurse	Undergraduate	Ward nurse
17	13	41	Head nurse	Postgraduate	Ward nurse
18	8	25	Nurse	Undergraduate	Emergency nurse
19	5	28	Nurse	Postgraduate	Surgical nurse
20	11	29	Nurse	Undergraduate	Surgical nurse

**Table 2:** Letters to experts.

Object	Years of work	Title	Academic qualifications	Specialities

1	7	Associate	Master's degree	Medical management
2	15	Full high	PhD	Nursing management
3	22	Senior	PhD	Medical management
4	30	Senior	PhD	Medical management
5	11	Associate	PhD	Nursing management
6	25	Deputy high	Master	Nursing management

**Table 3:** Overview of adverse events in nursing.

Category	Number	Proportion (%)

Nursing text recording errors	16	11
Drug allergy errors	10	7
Internship errors	7	5
Medication errors	22	15
Medication allergy errors	13	9
Slip of tubing	40	27
Other	37	26
Total	145	100

**Table 4:** Factors related to the quality of nursing safety management.

Category	Number	Proportion (%)

Nursing operations	86	59
Patient factors	39	27
Environmental factors	10	7
Instruments and equipment	3	2
Drugs and instruments	3	2
Other	4	3
Total	145	100

**Table 5:** Table of care.

Serial number	Projects	Evaluation		

1	Service attitude	Satisfied	Basic satisfied	Unsatisfied
2	Communication		*∗*	
3	Contraindications			*∗*
4	Operating techniques		*∗*	
5	Inspection		*∗*	
6	Timely assistance		*∗*	
7	Introduction to medication			*∗*
8	Dietary reminders			*∗*

## Data Availability

The data required in the article can be obtained from the corresponding author in the manuscript by e-mail.

## References

[1] Yan X., Zheng L. (2017). Fundamental analysis and the cross-section of stock returns: a data-mining approach. *Review of Financial Studies*.

[2] Wu W., Peng M. (2017). A data mining approach combining $K$ -means clustering with bagging neural network for short-term wind power forecasting. *IEEE Internet of Things Journal*.

[3] Gimeno B. A. (2017). Quality management, a directive approach to patient safety. *Enfermería Clínica (English Edition)*.

[4] Blenkinsopp J., Snowden N., Mannion R. (2019). Whistleblowing over patient safety and care quality: a review of the literature. *Journal of Health, Organisation and Management*.

[5] Ramos J., Castellanos-Garzón J. A., Depaz J. F., Corchado J. M. (2018). A data mining framework based on boundary-points for gene selection from DNA-microarrays: pancreatic Ductal Adenocarcinoma as a case study. *Engineering Applications of Artificial Intelligence*.

[6] Lin C.-J., Wu C., Chaovalitwongse W. A. (2015). Integrating human behavior modeling and data mining techniques to predict human errors in numerical typing. *IEEE Transactions on Human-Machine Systems*.

[7] Yang H.-H., Huang M.-L., Lai C.-M., Jin J.-R. (2018). An approach combining data mining and control charts-based model for fault detection in wind turbines. *Renewable Energy*.

[8] Cheng F., Fu X., Yan C. (2018). Research and applications of data mining techniques for improving building operational performance. *Current Sustainable/renewable Energy Reports*.

[9] Stalter A. M., Mota A. (2018). Using systems thinking to envision quality and safety in healthcare. *Nursing Management*.

[10] Leming-Lee T. S., Watters R., Watters R. (2019). Translation of evidence-based practice. *Nursing Clinics of North America*.

[11] Goedhart N. S., van Oostveen C. J., Vermeulen H. (2017). The effect of structural empowerment of nurses on quality outcomes in hospitals: a scoping review. *Journal of Nursing Management*.

[12] Coronado-Vázquez V., García-López A., López-Sauras S., Turón Alcaine J. M. (2017). Nursing involvement in risk and patient safety management in Primary Care. *Enfermería Clínica (English Edition)*.

[13] Sloane D. M., Smith H. L., Mchugh M. D., Aiken L. H. (2018). Effect of changes in hospital nursing resources on improvements in patient safety and quality of care. *Medical Care*.

[14] Tsai W.-P., Huang S.-P., Cheng S.-T., Shao K.-T., Chang F.-J. (2017). A data-mining framework for exploring the multi-relation between fish species and water quality through self-organizing map. *The Science of the Total Environment*.

[15] Grocott K. (2017). Quality and safety in nursing: a competency approach to improving outcomes sherwood gwen barnsteiner jane quality and safety in nursing: a competency approach to improving outcomes 424pp £45.99 wiley blackwell 9781119151678 1119151678. *Nursing Management*.

[16] Jie X., Reale C., Slagle J. M. (2017). Facilitated nurse medication-related event reporting to improve medication management quality and safety in intensive care units. *Nursing Research*.

[17] Zheng L., Hu W., Min Y. (2015). Raw wind data preprocessing: a data-mining approach. *IEEE Transactions on Sustainable Energy*.

[18] Rupesh W., Sagar J., Rahul S. (2017). An internal intrusion detection and protection system by using data mining and forensic techniques. *IEEE Systems Journal*.

[19] Marozzo F., Talia D., Trunfio P. (2018). A workflow management system for scalable data mining on clouds. *IEEE Transactions on Services Computing*.

[20] Xu L., Jiang C., Wang J. (2017). Information security in big data: privacy and data mining. *IEEE Access*.

[21] Buczak A. L., Guven E. (2016). A survey of data mining and machine learning methods for cyber security intrusion detection. *IEEE Communications Surveys & Tutorials*.

[22] Kavakiotis I., Tsave O., Salifoglou A., Maglaveras N., Vlahavas I., Chouvarda I. (2017). Machine learning and data mining methods in diabetes research. *Computational and Structural Biotechnology Journal*.

[23] Serdar M. A., Can B. B., Kilercik M. (2017). Analysis of changes in parathyroid hormone and 25 (OH) vitamin D levels with respect to age, gender and season: a data mining study. *Journal of Medical Biochemistry*.

[24] Moustakas A., Evans M. R. (2017). A big-data spatial, temporal and network analysis of bovine tuberculosis between wildlife (badgers) and cattle. *Stochastic Environmental Research and Risk Assessment*.

[25] Pourghasemi H. R., Yousefi S., Kornejady A., Cerdà A. (2017). Performance assessment of individual and ensemble data-mining techniques for gully erosion modeling. *The Science of the Total Environment*.

[26] Chaurasia V., Pal S. (2017). A novel approach for breast cancer detection using data mining techniques. *Social Science Electronic Publishing*.

[27] Huang Y., Li T., Luo C., Fujita H., Horng S.-j. (2017). Matrix-based dynamic updating rough fuzzy approximations for data mining. *Knowledge-Based Systems*.

[28] Akin M., Eyduran E., Reed B. M. (2017). Use of RSM and CHAID data mining algorithm for predicting mineral nutrition of hazelnut. *Plant Cell, Tissue and Organ Culture*.

[29] Emoto T., Yamashita T., Kobayashi T. (2017). Characterization of gut microbiota profiles in coronary artery disease patients using data mining analysis of terminal restriction fragment length polymorphism: gut microbiota could be a diagnostic marker of coronary artery disease. *Heart and Vessels*.

[30] Varley J. B., Miglio A., Ha V.-A., van Setten M. J., Rignanese G.-M., Hautier G. (2017). High-throughput design of non-oxide p-type transparent conducting materials: data mining, search strategy, and identification of boron phosphide. *Chemistry of Materials*.

